The article "Role of ErbB1 in the Underlying Mechanism of Lapatinib-Induced Diarrhoea: A Review" was published in 2022. Journal: Biomed Res Int.

# Role of ErbB1 in the Underlying Mechanism of Lapatinib-Induced Diarrhoea: A Review

**DOI:** 10.1155/2022/4165808

**Published:** 2022-06-28

**Authors:** Raja Nur Firzanah Syaza Raja Sharin, Jesmine Khan, Mohamad Johari Ibahim, Mudiana Muhamad, Joanne Bowen, Wan Nor I'zzah Wan Mohamad Zain

**Affiliations:** ^1^Department of Biochemistry and Molecular Medicine, Faculty of Medicine, Universiti Teknologi MARA, Sungai Buloh Campus, Jalan Hospital, 47000 Sungai Buloh, Selangor, Malaysia; ^2^Discipline of Physiology, School of Biomedicine, University of Adelaide, South Australia 5005, Australia

## Abstract

Lapatinib, an orally administered small-molecule tyrosine kinase inhibitor (SM-TKI), is an effective treatment for ErbB2-positive breast cancer. However, its efficacy as one of the targeted cancer therapies has been hampered by several adverse effects, especially gastrointestinal toxicity, commonly manifested as diarrhoea. Although it can be generally tolerated, diarrhoea is reported as the most common and most impactful on a patient's quality of life and associated with treatment interruption. Severe diarrhoea can result in malabsorption, leading to dehydration, fatigue, and even death. ErbB1 is an epidermal growth factor profoundly expressed in normal gut epithelium while lapatinib is a dual ErbB1/ErbB2 tyrosine kinase inhibitor. Thus, ErbB1 inhibition by lapatinib may affect gut homeostasis leading to diarrhoea. Nevertheless, the underlying mechanisms remain unclear. This review article provides evidence of the possible mechanisms of lapatinib-induced diarrhoea that may be related to/or modulated by ErbB1. Insight regarding the involvement of ErbB1 in the pathophysiological changes such as inflammation and intestinal permeability as the underlying cause of diarrhoea is covered in this article.

## 1. Introduction

Diarrhoea is a common gastrointestinal (GI) toxicity that is associated with a wide range of cancer treatments. In particular, receptor tyrosine kinase inhibitors (TKIs) directed against the epidermal growth factor receptor (EGFR) have diarrhoea as a class effect while diarrhoea induced by chemotherapy is not exclusively an epithelial effect but rather a complicated interaction between all mucosal compartments [1]. Nevertheless, no clinical guidelines are designed specifically for the management of TKIs-induced diarrhoea [2], contradictory to chemotherapy-induced diarrhoea which has several guidelines, including from the European Society for Medical Oncology (ESMO) and US National Comprehensive Cancer Centre Network [3]. This lack of clinical guideline was attributable to limited investigations on the underlying mechanisms of diarrhoea induced by targeted drugs. Thus, the treatment management of TKIs follows the management of chemotherapy-induced diarrhoea [4]. Although it can be abided, diarrhoea can affect about 50% to 80% of patients, depending on the treatment strategy [5].

The article "Role of ErbB1 in the Underlying Mechanism of Lapatinib-Induced Diarrhoea: A Review" was published in 2022. Journal: Biomed Res Int.

Severe diarrhoea can cause dehydration, malabsorption, fatigue, bowel discomfort, and perianal skin breakdown [6]. Furthermore, administration of small-molecule tyrosine kinase inhibitors (SM-TKIs) as cancer targeted therapies is prescribed for longer duration; thus, diarrhoea is often prolonged, which significantly compromises the quality of life (QOL) of patients with cancer. Indisputably so, effective treatment strategies for SM-TKIs-induced diarrhoea are critically needed, towards immediate identification of appropriate mechanisms of SM-TKIs-induced diarrhoea.

Lapatinib is an orally administered, dual ErbB1 and ErbB2 TKI and proven effective in treating ErbB2-positive breast cancer. Lapatinib reversibly binds to the intracellular adenosine triphosphate- (ATP-) binding site of the tyrosine kinase domain and prevents receptor phosphorylation and activation, hence blocking downstream signalling pathways such as mitogen-activated protein kinase/extracellular signal-regulated kinase (MAPK/Erk) and phosphatidylinositol-3′-kinases (PI3K)/Akt pathways which are involved in cell survival and proliferation, respectively [7]. In other words, the mechanism of action of lapatinib is by inhibition of ErbB1 and ErbB2 kinase activity, thus preventing the activation of downstream cellular signals that promote tumour cell survival and proliferation.

Despite its success as an ErbB2-positive breast cancer treatment, lapatinib has raised concern on gastrointestinal toxicity, specifically diarrhoea, which affects 78% of patients [8]. Several possible aetiologies have been hypothesised and discussed to account for lapatinib-induced diarrhoea. Leading theories investigated in preclinical models relate to alteration of chloride secretion and intestinal histopathological changes in the gastrointestinal tract (GIT) [8–10]; however, none of these studies were able to conclude a solid rationale for the mechanism of lapatinib-induced diarrhoea. Previous studies in particular have shown that inhibition of ErbB1 resulted in intestinal atrophy in mice by a loss of epithelial length [11], nutrient and electrolyte transport, and brush border enzyme expression [12]. Meanwhile, other studies using lapatinib in tumour-bearing models showed no evidence of histopathological changes at all, making this pathogenesis of diarrhoea remain unclear.

Thus, in this article, the possible underlying mechanisms of lapatinib-induced diarrhoea pertaining to ErbB1 involvement in inflammation and intestinal permeability based on *in vitro* and *in vivo* studies which may contribute to changes in intestinal health were discussed in detail. The associations between lapatinib and diarrhoea and how ErbB1 inhibition leads to intestinal inflammation and permeability were outlined. The inclusion criteria for the studies were (i) incidence of diarrhoea related to SM-TKIs, (ii) lapatinib gastrointestinal toxicity, and (iii) SM-TKIs affecting gastrointestinal changes from year 2005 to 2021, using the Boolean operator “AND.” The keywords used during the search were lapatinib and “diarrhea/diarrhoea”, EGFR/ErbB1 and “intestinal inflammation”, EGFR/ErbB1 and “intestinal permeability”, and EGFR/ErbB1 and “intestinal tight junction”. A total of 60 articles were included in this narrative review, while the rest were excluded due to repetitive experiments, review articles, and some articles being not totally related to the search topic.

The article "Role of ErbB1 in the Underlying Mechanism of Lapatinib-Induced Diarrhoea: A Review" was published in 2022. Journal: Biomed Res Int.

### 1.1. ErbB Family Receptors

The ErbB family of tyrosine kinase receptors are cell surface receptors, with four types of proteins which are EGFR/ErbB1/HER1, ErbB2/Neu/HER2, ErbB3/HER3, and ErbB4/HER4. All these proteins are important in regulating cell proliferation, differentiation, migration, and opposing cell death [13]. Each of the ErbB members exists as monomeric receptors [14]. Upon activation, these receptors can form ten different homodimers and heterodimers, initiating multiple signalling pathways such as ERK/protooncogene protein P21 (ERK/Ras), PI3K/Akt, phosphoinositide phospholipase C-*γ*1 (PLC*γ*1), and signal transducer and activator of transcription proteins/Src (STAT/Src) [15, 16].

ErbB2 does not contain a ligand-binding domain, yet ErbB2 appears to be the preferred binding partner to its family members, as its dimerization arm is constitutively exposed. ErbB3 does not contain a kinase domain; therefore, ErbB3 homodimers possess little autophosphorylation activity. However, ErbB3 can still be phosphorylated and induce potent downstream. ErbB1 on the other hand has six other ligands in addition to epidermal growth factor (EGF) which are transforming growth factor-alpha (TGF-*α*), amphiregulin (AREG), epiregulin (EREG), betacellulin (BTC), heparin-binding EGF-like growth factor (HB-EGF), and epigenin (EPI). Both ErbB1 and ErbB4 are targeted by BTC, HB-EGF, and EREG. Notably, another ErbB ligand, neuregulins (NRGs), can bind both ErbB3 and ErbB4 or only ErbB4 [17].

In healthy tissues, ErbB members are expressed in the brain, skin, lung, and GIT [17]. However, several studies have reported that overexpression of ErbB family members, especially ErbB2 either *in vitro* or *in vivo*, leads to cell transformation and metastasis [18]. Meanwhile, overexpression of ErbB1 has been correlated with gastric cancer, human hepatocellular carcinoma, and oesophageal cancer [19], and ErbB3 has been implicated in breast, bladder, and gastric cancers [13], whereas ErbB4 is also commonly associated with gastrointestinal cancer [20]. As such, inhibition of ErbB members and their downstream signalling provides a therapeutic option against human tumours with overexpression of ErbBs.

The article "Role of ErbB1 in the Underlying Mechanism of Lapatinib-Induced Diarrhoea: A Review" was published in 2022. Journal: Biomed Res Int.

Specifically, all these ErbBs can be found abundantly in small intestinal cells but have lower expression in Paneth cells [21]. However, a study using single-cell mapping showed no expression of ErbB4 throughout the epithelium [22], but both EGF and NRG1-expressing cells were identified in the developing human intestinal tract, with EGF being found in the epithelial villus domain and NRG1 being discovered in cells inside the subepithelial mesenchyme underneath the crypts [23].

ErbB1 promotes intestinal restitution/wound healing, cell survival, ion transport, and other essential elements of mucosal cell physiology. Reports comparing ligands with different receptor specificity define different outcomes. For example, ErbB1/ErbB4 ligands such as HB-EGF promote intestinal cell migration and proliferation, while NRG4 stimulates only cell survival [24]. Numerous studies especially *in vitro* and *in vivo* clearly concluded that ErbB1 activation necessitates protective responses in inflammatory bowel disease (IBD) models. Besides, the effects of probiotic organisms such as *Lactobacillus rhamnosus GG* against dextran-sulphate sodium- (DSS-) induced colitis also depend on ErbB1 activity. Similarly, activation of ErbB4 showed protective effects on the epithelium; for instance, intraperitoneal NRG4 administration blocks cytokine-induced colonocyte apoptosis and reduces histopathological damage in the DSS-induced colitis model. Loss of ErbB4, however, sensitizes epithelial cells to tumour necrosis factor-induced death [25].

The role of ErbB1 has also been studied extensively in the regulation and maintenance of the intestinal stem cell (ISC) niche. Several investigators showed that ErbB1 is crucial for ISC proliferation but not differentiation. In contrast, others reported that it does in fact involve both. However, a bacterial infection-induced injury study reported that ErbB1 is involved in differentiation and/or proliferation and cell shedding to remodel and maintain the homeostasis of the gut lining after the injury. This process perhaps involves reducing the cell number, shortening the gut and its elongation, increasing the number of differentiated cells, and then replenishing the ISC compartments in a nicely orchestrated manner at specified time points [26].

The article "Role of ErbB1 in the Underlying Mechanism of Lapatinib-Induced Diarrhoea: A Review" was published in 2022. Journal: Biomed Res Int.

In cultured intestinal cells, activation of ErbB promotes cellular outcomes that would be anticipated to be protective during inflammation. In colon epithelial cells, for example, ErbB1 increases proliferation, decreases cytokine-induced apoptosis, and promotes migration/wound healing both *in vitro* and *in vivo*. Specific ligand/receptor combinations can elicit selective responses; for example, NRG4, which selectively activates ErbB4, signals for mouse colonocyte survival but not proliferation or migration. This implies that with a greater knowledge of the relative effects of various ligands and receptors, a substantial degree of selectivity in response may be gained [27].

Both ErbB2 and ErbB3 are detected throughout the crypt-villus axis [22]. Determination of ErbB2 and ErbB3 roles in the intestine has been augmented by numerous studies, with various hypotheses being reached. Although no ligands have been identified for ErbB2, its activation can be induced by heterodimerization with ligand-occupied ErbB1, ErbB3, or ErbB4. ErbB2 has been implicated in mediating myoblast cell survival and in inhibiting cancer cell apoptosis [17]. In addition, ErbB2 has been shown to be transactivated by tumour necrosis factor-alpha (TNF-*α*), which in turn protects intestinal epithelial cells from TNF-*α*-induced apoptosis.

Even though ErbB3 homodimers possess little autophosphorylation activity, however, ErbB3 is often overexpressed in colorectal cancers when associated with ErbB1 and ErbB2. Intestine-specific ErbB3 ablation showed more damage to colonic epithelial cells and slow recovery of epithelial cells in a model of colitis induced by dextran sulphate sodium (DSS) [28]. Moreover, in a mutant allele of murine Apc (*adenomatous polyposis coli*) (*Apc^Min^*) intestinal tumour mouse model, intestine-specific ErbB3 knockout mice have less cellular proliferation within polyps in the intestine than the control mice [28].

### 1.2. ErbB1 Inhibition as Targeted Therapeutic for Cancer

ErbB1/EGFR/HER1 is a 170 kDa transmembrane glycoprotein that is composed of a single polypeptide chain and can either form homodimers or heterodimers with other ErbB members, ErbB2, ErbB3, and ErbB4. It has the largest number of signalling which includes ERK/MAPK, PI3K/Akt, SRC, PLC*γ*1/PKC, JNK, and JAK/STAT pathways [13], thus generating various diversity of cellular responses including cell proliferation, differentiation, apoptosis, and mortality [29]. Nonetheless, overexpression of ErbB1 was elucidated in several cancers such as colon, breast, and brain [30], rendering blockage of ErbB1 as a viable therapeutic option for the treatment of those tumours.

The article "Role of ErbB1 in the Underlying Mechanism of Lapatinib-Induced Diarrhoea: A Review" was published in 2022. Journal: Biomed Res Int.

ErbB1 targeted therapies can be divided into monoclonal antibodies (mAbs) and single-targeted TKIs, dual-targeted TKIs, and multitargeted TKIs (generally known as SM-TKIs). mAbs that have been authorised for clinical use include cetuximab, panitumumab, nimotuzumab, and necitumumab, which are intended to selectively attach to the epitopes expressed on tumour cells in a distinct manner [31]. Specifically, they were generated against the ErbB1 receptor's ligand-binding extracellular domain and compete with ErbB1 ligands such as EGF to inhibit phosphorylation and activate ErbB1-associated kinases [31]. As such, these will inhibit cellular growth and activation of apoptosis and decrease the growth factor production [32]. In addition, mAb is reported to have a higher affinity towards ErbB1 and possesses a longer half-life (e.g., 7.5 days for panitumumab) compared to SM-TKI (e.g., 48 hours for gefitinib) [33], making it more potent as an ErbB1 inhibitor. The drugs are administered intravenously.

In contrast, SM-TKIs are designed to bind directly to the ATP-binding site in the kinase domain of ErbB1 receptors and abolish their intracellular kinase activity [34]. Single-target TKIs such as gefitinib and erlotinib could bind only one tyrosine kinase inhibitor. Lapatinib a dual-target TKI pursues ErbB1 and ErbB2 simultaneously, thus indirectly inhibiting both phosphorylation and downstream signal transduction such as PI3K and MAPK pathways [35]. Additionally, multitargeted TKI drugs such as afatinib and dacomitinib target several tyrosine kinase receptors simultaneously through inhibition of cell proliferation and differentiation such as PLC*γ* and Wnt pathways [36]. Even though SM-TKIs have a short half-life, these orally active agents are suitable for long-term therapy.

Noted that, all these TKIs also differ in terms of their pharmacokinetics, which depends on the drug absorption, metabolization, and distribution and can be affected by pharmacogenetic of patients' background [33]. It is imperative to state that the distribution and metabolism between SM-TKIs and mAbs showed different mechanisms and molecular characteristics. Panitumumab, for instance, is administered at 6 mg/kg every 2 weeks, with typical absolute systematic availability of 70% [37]. It is mainly distributed into vascular space, which is able to prolong survival in patients with metastatic colorectal cancer. Meanwhile, the typical absolute systemic availability following oral treatment is 103.8% [38]. Gefitinib is likely to pass the blood-brain barrier, which might be beneficial in individuals with metastatic illness. It reaches steady-state concentrations in about 10 days. In short, SM-TKI is rapidly absorbed and distributed in large amounts (volume of distribution (Vd) > 100 L) compared to mAb which is distributed to the tissue slowly due to its large size (Vd < 10 L) [39]. In terms of metabolism, cytochrome P450 (CYP) 3A4 is primarily responsible for the SM-TKI oxidation and reduction process which resulted in renal elimination in urine and conjugation processes leading to hepatic/biliary elimination in the stool [40]. Meanwhile, mAbs are degraded into peptides and amino acids by circulating phagocytic cells or their target antigen-containing cells [41]. All of these contribute to a plausible reason for less severity of GI toxicity in mAbs compared to SM-TKIs. However, SM-TKIs have a notable benefit over mAbs in that they are available orally and allow for more convenient administration as compared to intravenous infusion, which requires outpatient visits.

The article "Role of ErbB1 in the Underlying Mechanism of Lapatinib-Induced Diarrhoea: A Review" was published in 2022. Journal: Biomed Res Int.

### 1.3. Incidence of Diarrhoea Associated with ErbB1 Targeted Drugs

Diarrhoea has been reported as the most common side effect of ErbB1 targeted SM-TKI agents after rash and frequently affects the rapidly dividing cells of the intestinal epithelium. It can be debilitating and lead to life-threatening adverse effects when it occurs in combinations with other complications such as neutropenia and cardiovascular morbidity [42]. Diarrhoea occurs approximately on day 7 of the treatment period, especially for multi-ErbB SM-TKI, with a common presentation of mild diarrhoea (grade 1-2). Noted that, mild diarrhoea should be considered an imperative case as prolonged diarrhoea affects patients' QOL. A previous clinical study using neratinib, an example for multi-ErbB SM-TKI, has shown that about 40% of severe diarrhoea (grade 3-4) incidence has been reported among 1408 patients. Meanwhile, lapatinib-induced diarrhoea showed a higher percentage among other first-generation TKIs, about 25% (Table 1). Diarrhoea can be caused by ErbB inhibitors alone or related to the combination treatment with chemotherapy. Furthermore, recent clinical studies have shown that all grades of diarrhoea are more commonly seen with second-generation pan-ErbB SM-TKIs rather than first-generation ErbB SM-TKIs. Even though it can be said that single-target TKIs would offer a greater chance of treatment compared to other multitargeted TKIs, it might be limited to this statement of whether all kinases have equal contribution to carcinogenesis [43]. Besides, there is a possibility that some receptor tyrosine kinases in healthy cells would also be inhibited by these multi-TKIs due to their unspecific TKI binding [43], thus leading to a new concern on classical toxicities of these compounds such as diarrhoea, rashes, and, even worse, cardiovascular toxicity [44]. In general, understanding of the TKIs-induced diarrhoea mechanism allows a cautious optimism to further enrich the therapeutic armamentarium against this side effect, hence improving the QOL of patients with cancer.

The article "Role of ErbB1 in the Underlying Mechanism of Lapatinib-Induced Diarrhoea: A Review" was published in 2022. Journal: Biomed Res Int.

### 1.4. Treatment of Diarrhoea Associated with ErbB1 Targeted Drugs

In general, management of cancer therapy-adverse effects (AEs) should consist of prophylactic measures, supportive medications, treatment delays, and dose reductions. The American Society and Clinical Oncology (ASCO) together with the European Society for Medical Oncology (ESMO) have established several consensus guidelines for cancer treatment-induced diarrhoea. The approach to diarrhoea management is based on severity and complication level, which includes hospital admission and self-administered antidiarrhoeal agents such as loperamide and octreotide to regulate gut motility and administration of intravenous fluids [58]. Loperamide is a synthetic opioid which agonizes opioid receptors present in the gastrointestinal tract [59]. There are several mechanisms of action of loperamide which reduce the peristalsis, increase gut transit time, and promote fluid absorption. Loperamide can be considered a conventional diarrhoea treatment; however, the efficiency as the first-line therapy for diarrhoea patients has been associated with other consequences, such as severe constipation and nausea [3]. Besides, prolonged use of high doses of loperamide for diarrhoea treatment can cause prolonged corrected QT interval (QTc) and provoke life-threatening arrhythmias, such as ventricular fibrillation [60]. Thus, octreotide becomes the second choice when loperamide fails. This can be a plausible merit to investigate new target treatments for ErbB1 TKI-induced diarrhoea. However, targeting interventions that effectively prevent or manage ErbB1 TKI-induced diarrhoea can only be achieved by understanding the underlying mechanisms.

### 1.5. Roles of ErbB1 in the Possible Mechanisms of Lapatinib-Induced Diarrhoea

#### 1.5.1. Lapatinib

Lapatinib (GW-572016) is a novel member of the 4-anilinoquinazoline class of kinase inhibitors which consist of a large aniline quinazoline head group, thus enhancing deep access into the catalytic cleft of ErbB1 [2]. The drug reversibly binds to the intracellular ATP-binding cytoplasmic domain of tyrosine kinase receptor thus blocking the receptor leading to activation of certain pathways including PI3K/Akt, MAPK [61], and PLC*γ* by decreasing the phosphorylation of the targeted receptor and Raf, Erk, Akt, and PLC*γ*1 proteins [62]. Lapatinib is a potent, reversible, and selective dual inhibitor of EGFR and ErbB2 kinases [63]. Xiang et al. reported the half-maximal inhibitory concentration (IC_50_) of lapatinib in nineteen tumour cells of gastric cancer, melanoma, hepatocarcinoma, thyroid, breast, pancreatic, and colorectal cell lines. This study revealed that proliferation IC_50_ values were <8 *μ*M, showing different degrees of lapatinib sensitivity. All these cell lines were then divided into two groups, high-IC_50_ and low-IC_50_ by taking 8 *μ*M of IC_50_ as the threshold to observe the ErbB1 and ErbB2 expression. It was noted that expression of ErbB1 and ErbB2 was significantly higher in the low-IC_50_ group (IC_50_ < 8 *μ*M), thus concluding that lapatinib sensitivity is positively correlated with the ErbB pathway [64]. Lapatinib was approved by the Food and Drug Administration (FDA) in 2007, as a second line for ErbB2 metastatic breast cancer, along with capecitabine [65], a prodrug of fluorouracil which has high absorption in GIT [66]. The approved dose for lapatinib is 1,250 mg per day, five 250 mg tablets per day taken continuously along with capecitabine 2,000 mg/m^2^ per day during days 1–14 of each 21-day treatment cycle [4].

The article "Role of ErbB1 in the Underlying Mechanism of Lapatinib-Induced Diarrhoea: A Review" was published in 2022. Journal: Biomed Res Int.

#### 1.5.2. Lapatinib and Diarrhoea

Like other TKIs, lapatinib does not just impose diarrhoea [12, 61, 67, 68], along with hypertension [67] and rash that tends to be localized most frequently on the trunk but infrequently on the face [2]. Although diarrhoea seems common, it is often severe enough to require a break in treatment or a dose reduction [6]. Diarrhoea in lapatinib administration was evident as early as 7 days of the treatment course and has been managed usually with antidiarrhoeal agents depending on the treatment protocol [69]. However, it is hypothesised that the development of lapatinib-induced diarrhoea differs from conventional chemotherapy-induced diarrhoea and is not due to direct cytotoxicity but through alternative mechanisms [70]. Thus, traditional diarrhoea management may not be targeting the underlying changes for optimal management.

Various hypotheses have been reported regarding the underlying mechanism of lapatinib-induced diarrhoea such as alteration of chloride secretion in the gut lumen and changes in gut microflora, and the most notable theory is inhibition of ErbB1 in gastrointestinal mucosa. ErbB1 is expressed in GI mucosa which is the primary site for the drug absorption in the intestine. Thus, the administration of ErbB1 SM-TKI may interfere with normal functioning, leading to diarrhoea.

One such hypothesis theorized that diarrhoea from ErbB SM-TKIs is a form of secretory diarrhoea, activated by apical chloride channels such as calcium-activated chloride channels (CaCC) and cystic fibrosis transmembrane conductance regulator (CFTR) [71]. In this mechanism, the chloride channels increase the fluid secretion into the lumen, thereby inhibiting the absorption of intestinal sodium, which reduces overall fluid absorption. It has been reported that ErbB1 has an inhibitory effect on chloride secretion in the small intestine, which raises the hypothesis that inhibition of ErbB1 in the intestine allows the excessive chloride secretion into the gut lumen. An *in vitro* study has evidenced that dacomitinib, a pan-ErbB TKI, increased intestinal epithelial chloride secretion [72]. Moreover, previous studies using an *in vivo* model on dacomitinib and neratinib-induced diarrhoea suggested that the diarrhoea was secretory in nature. However, treatment with an antidiarrhoeal agent, crofelemer, which is also an antichloride secretory medication on *in vivo* model-induced dacomitinib worsened diarrhoea levels [73]. Studies on chloride secretion following lapatinib and neratinib in a rat model show no evidence of change, thus leaving the role of chloride secretion unclear [53, 70] with major discordance in findings between *in vitro* and *in vivo* settings.

The article "Role of ErbB1 in the Underlying Mechanism of Lapatinib-Induced Diarrhoea: A Review" was published in 2022. Journal: Biomed Res Int.

Aside from ErbB1-induced alterations in chloride secretion, direct damage to the GI mucosa by the oral administration of ErbB1 SM-TKIs has been reported. Studies using ErbB1 knockout mice and other ErbB1 SM-TKIs have described mucosal atrophy supporting a role for direct mucosal damage [74, 75]. Besides inhibiting tumour cell survival and proliferation, ErbB1 SM-TKIs are also said to inhibit the normal function of ErbB1 in the gastrointestinal mucosa. This is shown by a study by Secombe et al. who found decreased activation of ErbB1 in rat models after treatment with neratinib [76]. A recent study also has shown that ErbB1 SM-TKI-induced diarrhoea resulted from histopathological damage which was evidenced by significant growth reduction and villi atrophy in the ileum [72]. In contrast, studies using lapatinib in tumour-bearing models did not show any histopathological changes [70], thus making the mechanism of ErbB1 inhibition-induced diarrhoea unclear.

Besides the above hypotheses, another impetus for further investigation is whether ErbB1 SM-TKIs cause inflammation. A study using a TKI-induced diarrhoea model in 2019 has proved a decrease in diarrhoea incidence following neratinib when rats were treated with budesonide and colesevelam, in which both are used as anti-inflammatory agents in gastrointestinal conditions [76]. This result then was supported by increasing levels of interleukin-4 (IL-4), an anti-inflammatory interleukin in both the colon and ileum of budesonide-treated rats. In addition, there are also increased responses of inflammatory cytokines such as interferon-alpha (IFN-*α*) and interferon-gamma (IFN-*δ*) observed in both *in vitro* and tumour-bearing models treated with osimertinib [77]. One study by Lacouture et al. revealed that panitumumab-treated patients were able to suppress diarrhoea incidence to 56% compared to the reactive arm (85%) when administered with doxycycline as an antidiarrhoeal agent [78]. Note that doxycycline, an antibiotic, exhibited anti-inflammatory properties. Even though this is not a direct study of TKI-diarrhoea-induced inflammation, Lacouture et al. [78] later suggested that diarrhoea induced by ErbB1 might involve an inflammation process.

The article "Role of ErbB1 in the Underlying Mechanism of Lapatinib-Induced Diarrhoea: A Review" was published in 2022. Journal: Biomed Res Int.

A study by Leech et al. in 2018 on lapatinib-treated cells showed lower expression of junction adhesion molecule-A (JAM-A), a tight junction protein (TJP) that is highly expressed in normal epithelial and endothelial cells. This showed that administration of lapatinib does increase intestinal permeability by compromising TJP integrity [79] Additionally, an increase in permeability initiates recruitment of lipopolysaccharides (LPS) from the small intestinal lumen, promoting inflammatory cytokines to stimulate an immune reaction, thus activating inflammatory reaction [80]. These studies showed that lapatinib might induce diarrhoea by increasing the permeability of intestinal TJPs, thereby promoting inflammation.

In a dacomitinib-induced diarrhoea rat model, cytoplasmic redistribution of claudin-1 was seen in the ileum of the drug-treated rats, where peak histopathological damage such as blunting and villi fusion were observed. Inflammatory infiltrate was also noted in the ileum suggesting that the tight junction dysfunction can be proinflammatory cytokine-mediated [73]. Tumour necrosis factor-alpha (TNF-*α*), interleukin- (IL-) 1, and IL-6 also have been shown to contribute to the severity and degree of injury in chemotherapy-induced gut toxicity [81]. These studies emphasized the importance of the integrity of the structure and function of tight junction proteins of intestinal epithelial cells in the downstream signalling of ErbB1. As such, it is said that inflammation may impact the tight junctions which are also potential mechanisms leading to the diarrhoea in ErbB1 TKI-treated patients. Another potential avenue that could be associated with the oral-administered drug is the accumulation of unabsorbed drugs in the lumen due to its low bioavailability, thus leading to mucus secretion and therefore resulting in the osmotic movement of water in diarrhoea [82].

Based on this previous literature, the complex relationship between compromised gut wall integrity and mucosal inflammation has sparked scientific interest in various inflammatory bowel studies. However, it is unclear whether a damaged mucosal barrier promotes intestinal inflammation or whether poor barrier function is a side effect of the inflammatory process. Nonetheless, there is a well-established relationship between increased intestinal permeability and increased inflammatory activity.

The article "Role of ErbB1 in the Underlying Mechanism of Lapatinib-Induced Diarrhoea: A Review" was published in 2022. Journal: Biomed Res Int.

Together, these studies provide important insights to further enrich the understatement of lapatinib-induced diarrhoea mechanism. A conceptual framework was constructed (Figure 1) directing the concept that once administered, lapatinib binds to the intracellular ATP-binding site of the tyrosine kinase domain and inhibits receptor phosphorylation and activation. The drug then not only inhibits tumour cell survival and proliferation but also inhibits ErbB1 function in the GI mucosa. Inhibition of ErbB1 function disrupts gut homeostasis causing inflammation to the intestinal monolayer which leads to disruption of TJPs further adding to increased intestinal permeability, hence diarrhoea.

#### 1.5.3. ErbB1 and Inflammation in TKIs-Induced Diarrhoea

Inflammation is known as one of the key roles in the development of gastrointestinal problems, in which it is also believed to be involved in SM-TKIs-induced diarrhoea. Development of SM-TKIs-induced diarrhoea is said to differ from conventional chemotherapy-induced diarrhoea (CID) since it does not involve direct cytotoxicity [70, 72]. Thus, in the literature on SM-TKIs-induced inflammation, the relative importance of chemotherapy-induced inflammation has been subjected to considerable discussion.

Several studies have documented that the chemotherapy-induced diarrhoea mechanism involves regulation of 5-fluorouracil (5-FU), irinotecan, and its active metabolite, 7-ethyl-10-hydroxycamptothecin (SN38) [3]. Histological intestinal damage such as blunting villi, crypt ablation, and excessive mucus secretion [83] in a mouse model was evidenced from CID. It is also strongly believed that CID is associated with GI mucositis which can be divided into 5 sequential phases: initiation, upregulation, signalling and amplification, ulceration and inflammation, and healing [3]. In this context, the initiation phase involves initiation injury to tumour cells caused by chemotherapy and radiation, either directly through DNA damage or, more common, indirectly through reactive oxygen species. This causes a cascade of enzyme and transcription factor activation (e.g., nuclear factor, NF-*κβ*), which leads to the activation of inflammatory cytokines such as TNF-*α*, IL-1, and IL-6, which resulted in tissue damage in submucosa and basal epithelium, hence leading to ulceration and bacterial colonisation, perpetuating a vicious cycle of inflammatory cytokine-mediated harm [84]. This will eventually thin the mucosal barrier, which allows bacterial translocation and malabsorption thus resulting in diarrhoea [5]. The healing phase then involves signalling via the extracellular matrix which stimulates epithelial proliferation and epithelization, as such reestablishing the mucosal barrier. In addition, the latest study by Wardill et al. showed that activation of toll-like receptor (TLR) by irinotecan also attenuates the upregulation of the inflammation process in CID [85]. As such, CID is described to have a direct tissue damage mechanism, which differs from SM-TKIs that might involve indirect biological signalling.

The article "Role of ErbB1 in the Underlying Mechanism of Lapatinib-Induced Diarrhoea: A Review" was published in 2022. Journal: Biomed Res Int.

Recent studies of ErbB1 TKIs reported that mouse intestinal atrophy was evidenced through shortening of epithelial length in the intestine [11] and villi blunting with inflammatory infiltrate present in lamina propria [76], goblet cell depletion, and vacuolization [86]. Besides, a study on gefitinib and icotinib on IEC-6 cells also showed a significant increment in the expression of proinflammatory IL-6 and IL-25 [87]. However, another study using gefitinib showed that ErbB1 ablation in a mouse model of colitis had significantly downregulated the production of IL-33, an inflammatory cytokine in the intestine [88]. An *in vitro* model using dacomitinib also showed increased monocyte chemoattractant protein-1 (MCP1) expression in the ileum, which is an intestinal region in which ErbB1 expression was reported higher in this study [72]. A downstream study on knockdown of RHBDF2 gene which involves in activation of the ErbB1 pathway and is responsible for inflammation development in the IL-10-deficient mouse model of colitis displayed intestinal epithelial damage, with elevated neutrophil in the gut [89]. In addition, Xiao et al. proved that LPS-challenged piglets have lower mRNA expression of ErbB1 in the jejunal mucosa region, which strongly supported the correlation activity of downregulation of ErbB1 signalling initiating inflammatory responses [90]. However, such expositions are further required to demonstrate a link between ErbB1 inhibition and intestinal inflammation in lapatinib-induced diarrhoea.

#### 1.5.4. ErbB1 and Intestinal Permeability in TKIs-Induced Diarrhoea

The correlation between ErbB1 and intestinal permeability has been extensively studied, with solid conclusion that activation of ErbB1 signalling adorned intestinal barrier formation through elevated expression of tight junction proteins (TJPs) (claudins, occludins, junctional adhesion molecule-A (JAM-A), and zonula occludens (ZO)), mucin secretion, and enterocyte proliferation enhancement [91]. A healthy intestinal epithelium acts as a barrier which inhibits the permeation of proinflammatory chemicals such as infections and antigens from the luminal environment into mucosal tissue [92]. Disruption of the intestinal barrier, followed by luminal noxious molecule permeability, causes a disruption of the mucosal immune system and inflammation, which can serve as a trigger for the development of intestinal illnesses such as IBD and Crohn's disease. It is worth highlighting that increased intestinal paracellular permeability was identified as one of the main factors for these fiasco diseases [93, 94].

The article "Role of ErbB1 in the Underlying Mechanism of Lapatinib-Induced Diarrhoea: A Review" was published in 2022. Journal: Biomed Res Int.

Tight junctions (TJs) are acknowledged as incredibly dynamic structures that participate in several vital functions of the intestinal epithelium under both normal and pathological settings. Previous studies on ErbB1 signalling have proved to be dependent on TJ formation. For instance, a study using pretreatment of Caco-2, a colon adenocarcinoma cell with EGF, showed a redistribution of TJPs, ZO-1, and occludin, while inhibition of MAPK/Erk has totally abolished the protective effects of EGF on tight junctions (TJs) [95]. Noted here, EGF is a ligand that binds to the ErbB1 receptor, which leads to autophosphorylation activity of receptor tyrosine kinase (RTK) and activation of the downstream pathway of MAPK/Erk and PI3K/Akt, thus stimulating intestinal development [96]. In addition, EGF is mentioned to be a critical regulator of intestinal paracellular permeability, which is dependent on TJs [92]. In this context, inhibition of ErbB1 is stipulated to have an impact on impairment of TJ functions, as this would enhance the invasion of foreign substances into the body and further leakage in intestinal epithelial due to excessive bacterial antigens, thus triggering inflammatory responses [97–99]. This statement is supported by a study using SM-TKI, erlotinib that attenuated paracellular permeability and intestinal atrophy in a gliadin-administered mouse model, accompanied by inhibition of ErbB1 phosphorylation [80]. Administration of simotinib in a Caco-2 model also had reduced expression of afadin-6, a target protein for the ErbB1/Ras/MAPK signalling pathway that interacts with ZO-1 [100]. Furthermore, in another study using intestinal ischemia/reperfusion injury rats, administration of HB-EGF, known as ligand of ErbB1 and ErbB4 in this model, had significantly decreased the intestinal permeability by downregulating proinflammatory markers such as TNF-*α*, IL-6, and IL-1*β* [101]. This strongly proved the ability of ErbB1 signalling to protect the intestinal barrier by regulating inflammatory cytokine levels. Besides, exposure of Caco-2 cells to IFN-*γ*, IL-17A, and zonulin, a protein modulator in the small intestine that rapidly promotes intestinal permeability, demonstrated modification of TJP (ZO-1, claudin-5, and occludin) localization, followed by significant depolymerization of perijunctional F-actin cytoskeleton [102]. An interesting study by Tripathi et al. showed that zonulin, a precursor of haptaglobin-2 (pre-HP2), mediates the transactivation of ErbB1 via protease-activated receptor 2 (PAR2). This couple (pre-HP2/PAR2) modulates the increment in intestinal permeability. At ≥15 *μ*g/mL, single-chain zonulin is able to increase phosphorylation of ErbB1. As such, an *in vitro* validation test on Caco-2 cells with AG1478 and ErbB1 inhibitor prevented zonulin-induced ErbB1 phosphorylation as well as abolished reduction in transepithelial electrical resistance (TEER) of Caco-2 cells. In addition, zonulin digestion by trypsin dramatically hampered its ability to activate ErbB1 signalling [103]. This study proves that single-chain zonulin, not in its cleaved mature forms, activated ErbB1 through indirect transactivation via PAR2, which initiated TJ disassembly, thus reducing TEER in Caco-2 cells.

The article "Role of ErbB1 in the Underlying Mechanism of Lapatinib-Induced Diarrhoea: A Review" was published in 2022. Journal: Biomed Res Int.

Considering all these studies, inhibition of ErbB1 in the intestine by lapatinib is believed to trigger intestinal mucosal damage as well as initiate inflammatory response, together with nutrient malabsorption and histopathological changes. These factors then lead to an increase in intestinal permeability, with such barrier dysfunction having compromised intestinal epithelial TJs in the intestinal epithelium, resulting in diarrhoea. As such, there is abundant room for further progress in validating this hypothesis of lapatinib-induced diarrhoea.

### 1.6. Future Directions on Lapatinib-Induced Diarrhoea

Several preliminary *in vitro* and *in vivo* models were developed to further clarify the mechanism of diarrhoea related to lapatinib, with various alternative therapeutics having been introduced. However, the aetiology is still unclear with various hypotheses having been discovered related to the GI injury. This review represents the importance of ErbB1 inhibition caused by lapatinib as the most plausible hypothesis to anticipate this GI toxicity. Future research is needed with further deliberation on developing models that incorporate ErbB1 as an imperative indicator of SM-TKI treatment responses.

EGF, as mentioned before, is one of the prominent ligands that activate ErbB1 pathways and has been identified to exhibit a remarkable ability on protecting intestinal epithelium through stimulation of several underlying mechanisms. It is said to be a potent stimulator for epidermal and epithelial cell proliferation [104], regulating cell survival, migration, differentiation, and apoptosis [105]. Besides, EGF is heat-stable [91] and trypsin-resistant [106] and resistant to proteolytic degradation [105], thus making it suitable to be administered through the orogastric route [91]. Recent studies showed that EGF also functions as a gastrointestinal mucosal trophic agent and cryoprotective barrier [107], and its proliferative effect is able to be preserved despite the loss of epidermal growth factor receptor (EGFR) at enterocytes [105]. Moreover, secretion of EGF protein produced by recombinant *E. coli* Nissle 1917 acts as an in vitro wound healing agent and hastens epithelial migration activity in injured human enterocyte monolayers through activation of the ERK pathway [108]. In short, it is possible to say that cotreatment of lapatinib with recombinant ErbB1 ligands such as EGF would be able to prove whether ErbB1 alteration plays an important role in lapatinib action that leads to side effects such as diarrhoea.

The article "Role of ErbB1 in the Underlying Mechanism of Lapatinib-Induced Diarrhoea: A Review" was published in 2022. Journal: Biomed Res Int.

Taken together, these findings might suggest that EGF could be a predictive target for future development of clinical models to uncover the true causation of diarrhoea and hence might be the appropriate therapeutic approach. Though it is apparent that much more must be known about TKI-induced diarrhoea, with persistent study effort, future management of this side effect will be improved vastly.

## 2. Conclusion

Diarrhoea may seem manageable for a healthy person. However, it can aggravate cancer patients' QOL as well as compromise their treatment course. Therefore, effective prevention and precise treatment are imperative to reduce the burden of diarrhoea among cancer patients. In this article review, we have discussed the involvement of ErbB1 in SM TKIs-induced diarrhoea, especially by lapatinib, an oral HER2-positive breast cancer treatment. Even though previous research has speculated several hypotheses in the pathogenesis of SM TKIs-induced diarrhoea, we hypothesise that inhibition of ErbB1 in a normal intestine may play a role in this gastrointestinal toxicity. It is worth highlighting that there is still obscurity as to whether increased intestinal permeability is a result of the inflammatory response or a pathophysiologic predictor of disease. It is hoped that determining whether excessive intestinal permeability is the product of a continuing inflammatory response or whether the intestinal barrier function contributes to the diarrhoea progression will be critical to our knowledge of LID pathophysiology. As such, understanding of this mechanism would provide new insights and new directions to prevent and minimize the incidence subsequently towards novel intervention for diarrhoea prevention and improving patient's QOL.

The article "Role of ErbB1 in the Underlying Mechanism of Lapatinib-Induced Diarrhoea: A Review" was published in 2022. Journal: Biomed Res Int.

## Figures and Tables

**Figure 1:** Conceptual framework of the underlying mechanisms of lapatinib-induced diarrhoea. Treatment with lapatinib not only inhibits tumour cell survival and proliferation but also inhibits ErbB1 normal function in gastrointestinal mucosa (1). ErbB1 inhibition is hypothesised to disrupt gut homeostasis (2) by triggering excessive leakage of LPS or bacterial antigens into the mucosa, causing upregulation of inflammatory cytokines (3) that progressively destroys the intestinal epithelium, subsequently permitting more antigen leakage, aggravating inflammation responses thus compromising intestinal barrier permeability by altering intracellular TJPs (4 and 5), hence diarrhoea. Abbreviation: LPS: lipopolysaccharide; TJPs: tight junction proteins.

**Table 1:** Comparison of incidence of diarrhoea in ErbB1 targeted therapies.

Type of ErbB1 TKI	Receptor binding	Target	Indication	Route of administration	Diarrhoea incidence		References
					All grades (%)	Severe grade 3-4 (%)	
*Monoclonal antibodies (mAbs)* Cetuximab (Erbitux®/C225)	Irreversible	Extracellular domain III of ErbB1	HNSCC, metastatic colorectal cancer	Intravenous	3%	1.7%	[45]
Panitumumab (Vectibix®)	Irreversible	Extracellular domain III of ErbB1	Metastatic colorectal cancer, solid tumours	Intravenous	20%	1.3%	[46]
Nimotuzumab (h-R3)	Irreversible	Competitive binding to extracellular domain III of ErbB1 (353–358) with ligand	HNSCC, metastatic pancreatic cancer, oesophageal cancer, gastric cancer	Intravenous	2.73%	0.91%	[47]
Necitumumab (Portrazza™)	Irreversible	Competitive binding to extracellular domain III of ErbB1 (384–409) with ligand	NSCLC, solid tumours	Intravenous	7%	2%	[48]
*First generation* Erlotinib (Tarceva®)	Reversible	ErbB1	NSCLC, pancreatic cancer	Oral	43.4%-69.2%	1%-17%	[49–51]
Gefitinib (Iressa®)	Reversible	ErbB1	NSCLC	Oral	35.7%-56%	1%-3.8%	[42, 50]
Lapatinib (Tykerb/Tyverb®)	Reversible	ErbB1, ErbB2	Breast cancer	Oral	58%-78%	23.3%-25%	[8, 52]
*Second generation* Neratinib (Nerlynx®)	Irreversible	ErbB1, ErbB2, ErbB4	ErbB2-positive breast cancer	Oral	95%	39.8%	[53]
Afatinib (Giotrif®)	Irreversible	ErbB1, ErbB2, ErbB3, ErbB4	NSCLC	Oral	42%-92.9%	10%-16%	[50, 54]
Dacomitinib (Vizimpro®)	Irreversible	ErbB1, ErbB2, ErbB4	NSCLC	Oral	87%	8%	[55]
*Third generation* Osimertinib (Tagrisso®)	Irreversible	T790M ErbB1 mutation	NSCLC	Oral	47%-58%	2%-3.3%	[42, 56]
Tucatinib (Tukys®)	Reversible	ErbB2	ErbB2-positive breast cancer	Oral	81%	12.5%	[57]

Abbreviation: HNSCC: head and neck squamous cell carcinoma; NSCLC: non-small-cell lung cancer; T790M: Threonine790Methionine mutation.

The article "Role of ErbB1 in the Underlying Mechanism of Lapatinib-Induced Diarrhoea: A Review" was published in 2022. Journal: Biomed Res Int.

## Abbreviations

5-FU: 5-Fluorouracil
AEs: Adverse effects
Apc: *Adenomatous polyposis coli*
AREG: Amphiregulin
ASCO: American Society and Clinical Oncology
ATP: Adenosine triphosphate
BRAT: Banana, rice, applesauce, and toast
BTC: Betacellulin
CaCC: Calcium-activated chloride channels
Caco-2: Colorectal adenocarcinoma cells
CFTR: Cystic fibrosis transmembrane conductance regulator
CID: Chemotherapy-induced diarrhoea
DSS: Dextran-sulphate sodium
EGF: Epidermal growth factor
EGFR: Epidermal growth factor receptor
EPI: Epigenin
EREG: Epiregulin
ERK/Ras: Extracellular signal-regulated kinase/protooncogene protein P21
ESMO: European Society for Medical Oncology
GI: Gastrointestinal
GIT: Gastrointestinal tract
HB-EGF: Heparin-binding EGF-like growth factor
HNSCC: Head and neck squamous cell carcinoma
IBD: Inflammatory bowel disease
IC_50_: Half-maximal inhibitory concentration
IEC-6: Intestinal epithelioid cell no. 6
IFN-*δ*: Interferon-gamma
IFN-*α*: Interferon-alpha
IL-1: Interleukin-1
IL-25: Interleukin-25
IL-33: Interleukin-33
IL-4: Interleukin-4
IL-6: Interleukin-6
ISC: Intestinal stem cells
JAM-A: Junction adhesion molecule-A
LPS: Lipopolysaccharide
mAbs: Monoclonal antibodies
MAPK/Erk: Mitogen-activated protein kinase/extracellular signal-regulated kinase
MCP1: Monocyte chemoattractant protein-1
NF-*κβ*: Nuclear factor
NRG1: Neuregulin-1
NRG4: Neuregulin-4
NRGs: Neuregulins
NSCLC: Non-small-cell lung cancer
PAR2: Protease-activated receptor 2
PI3K: Phosphatidylinositol-3′-kinases
PLC*γ*1: Phosphoinositide phospholipase C-*γ*1
Pre-HP2: Precursor of haptaglobin-2
QOL: Quality of life
RHBDF2: Rhomboid 5 homolog 2
SM-TKIs: Small molecule tyrosine kinase inhibitors
SN38: 7-Ethyl-10-hydroxycamptothecin
STAT/Src: Signal transducer and activator of transcription proteins/Src
T790M: Threonine790Methionine mutation
TEER: Transepithelial electrical resistance
TGF-*α*: Transforming growth factor-alpha
TJP: Tight junction protein
TJPs: Tight junction proteins
TJs: Tight junctions
TKIs: Tyrosine kinase inhibitors
TLR: Toll-like receptor
TNF-*α*: Tumour necrosis factor-alpha
Vd: Volume of distribution
ZO: Zonula occludens
ZO-1: Zonula occludens-1.
